This article has been retracted.

# Detecting phishing websites using machine learning technique

**DOI:** 10.1371/journal.pone.0258361

**Published:** 2021-10-11

**Authors:** Ashit Kumar Dutta

**Affiliations:** Department of Computer Science and Information System, College of Applied Sciences, Almaarefa University, Riyadh, Saudi Arabia; Qingdao University, CHINA

## Abstract

In recent years, advancements in Internet and cloud technologies have led to a significant increase in electronic trading in which consumers make online purchases and transactions. This growth leads to unauthorized access to users’ sensitive information and damages the resources of an enterprise. Phishing is one of the familiar attacks that trick users to access malicious content and gain their information. In terms of website interface and uniform resource locator (URL), most phishing webpages look identical to the actual webpages. Various strategies for detecting phishing websites, such as blacklist, heuristic, Etc., have been suggested. However, due to inefficient security technologies, there is an exponential increase in the number of victims. The anonymous and uncontrollable framework of the Internet is more vulnerable to phishing attacks. Existing research works show that the performance of the phishing detection system is limited. There is a demand for an intelligent technique to protect users from the cyber-attacks. In this study, the author proposed a URL detection technique based on machine learning approaches. A recurrent neural network method is employed to detect phishing URL. Researcher evaluated the proposed method with 7900 malicious and 5800 legitimate sites, respectively. The experiments’ outcome shows that the proposed method’s performance is better than the recent approaches in malicious URL detection.

## 1. Introduction

Phishing is a fraudulent technique that uses social and technological tricks to steal customer identification and financial credentials. Social media systems use spoofed e-mails from legitimate companies and agencies to enable users to use fake websites to divulge financial details like usernames and passwords [1]. Hackers install malicious software on computers to steal credentials, often using systems to intercept username and passwords of consumers’ online accounts. Phishers use multiple methods, including email, Uniform Resource Locators (URL), instant messages, forum postings, telephone calls, and text messages to steal user information. The structure of phishing content is similar to the original content and trick users to access the content in order to obtain their sensitive data. The primary objective of phishing is to gain certain personal information for financial gain or use of identity theft. Phishing attacks are causing severe economic damage around the world. Moreover, Most phishing attacks target financial/payment institutions and webmail, according to the Anti-Phishing Working Group (APWG) latest Phishing pattern studies [1].

In order to receive confidential data, criminals develop unauthorized replicas of a real website and email, typically from a financial institution or other organization dealing with financial data [2–4]. This e-mail is rendered using a legitimate company’s logos and slogans. The design and structure of HTML allow copying of images or an entire website [5]. Also, it is one of the factors for the rapid growth of Internet as a communication medium, and enables the misuse of brands, trademarks and other company identifiers that customers rely on as authentication mechanisms [6–8]. To trap users, Phisher sends "spooled" mails to as many people as possible. When these e-mails are opened, the customers tend to be diverted from the legitimate entity to a spoofed website.

There is a significant chance of exploitation of user information. For these reasons, phishing in modern society is highly urgent, challenging, and overly critical [9, 10]. There have been several recent studies against phishing based on the characteristics of a domain, such as website URLs, website content, incorporating both the website URLs and content, the source code of the website and the screenshot of the website [11]. However, there is a lack of useful anti-phishing tools to detect malicious URL in an organization to protect its users. In the event of malicious code being implanted on the website, hackers may steal user information and install malware, which poses a serious risk to cybersecurity and user privacy. Malicious URLs on the Internet can be easily identified by analyzing it through Machine Learning (ML) technique [12, 13]. The conventional URL detection approach is based on a blacklist (set of malicious URLs) obtained by user reports or manual opinions. On the one hand, the blacklist is used to verify an URL and on the other hand the URL in the blacklist is updated, frequently. However, the numbers of malicious URLs not on the blacklist are increasing significantly. For instance, cybercriminals can use a Domain Generation Algorithm (DGA) to circumvent the blacklist by creating new malicious URLs. Thus, an exhaustive blacklist of malicious URLs [14, 15] is almost impossible to identify the malicious URLs. Thusnew malicious URLs cannot be identified with the existing approaches. Researchers suggested methods based on the learning of computer to identify malicious URLs to resolve the limitations of the system based on the blacklist [16–18]. Malicious URL detection is considered a binary classification task with two-class predictions: malicious and benign. The training of the ML method consists of finding the best mapping between the d-dimensional vector space and the output variable [19–21]. This strategy has a strong generalization capacity to find unknown malicious URLs compared to the blacklist approach.

Recurrent Neural Network (RNN)—Long Short-Term Memory (LSTM) is one of the ML techniques that presents a solution for the complex real—time problems [22]. LSTM allow RNN to store inputs for a larger period [23]. It is similar to the concept of storage in computer. In addition, each feature will be processed according to the uniform distribution [24]. The combination of RNN and LSTM enables to extract a lot of information from a minimum set of data. Therefore, it supports phishing detection system to identify a malicious site in a shorter duration.

In comparison to most previous approaches, researchers focus on identifying malicious URLs from the massive set of URLs. Therefore, the study proposes Recurrent Neural Network (RNN) based URL detection approach. The objectives of the study are as follows:

1. To develop a novel approach to detect malicious URL and alert users.
2. To apply ML techniques in the proposed approach in order to analyze the real time URLs and produce effective results.
3. To implement the concept of RNN, which is a familiar ML technique that has the capability to handle huge amount of data.

The rest of the paper is organized as follows: Section 1 introduces the concept of malicious URL and objective of the study. The background of the study and related literature in detecting URL is discussed in section 2. Section 3 presents the methodology of the research. Results and discussion are presented in section 4. Finally, section 5 concludes the study with its future direction.

## 2. Research background and related works

Phishing attacks are categorized according to Phisher’s mechanism for trapping alleged users. Several forms of these attacks are keyloggers, DNS toxicity, Etc., [2]. The initiation processes in social engineering include online blogs, short message services (SMS), social media platforms that use web 2.0 services, such as Facebook and Twitter, file-sharing services for peers, Voice over IP (VoIP) systems where the attackers use caller spoofing IDs [3, 4]. Each form of phishing has a little difference in how the process is carried out in order to defraud the unsuspecting consumer. E-mail phishing attacks occur when an attacker sends an e-mail with a link to potential users to direct them to phishing websites.

### 2.1 Classification of phishing attack techniques

Phishing websites are challenging to an organization and individual due to its similarities with the legitimate websites [5]. Fig 1 presents the multiple forms of phishing attacks. Technical subterfuge refers to the attacks include Keylogging, DNS poisoning, and Malwares. In these attacks, attacker intends to gain the access through a tool / technique. On the one hand, users believe the network and on the other hand, the network is compromised by the attackers. Social engineering attacks include Spear phishing, Whaling, SMS, Vishing, and mobile applications. In these attacks, attackers focus on the group of people or an organization and trick them to use the phishing URL [6, 7]. Apart from these attacks, many new attacks are emerging exponentially as the technology evolves constantly.

**Fig 1:** Multiple forms of phishing attacks.

### 2.2 Phishing detection approaches

Phishing detection schemes which detect phishing on the server side are better than phishing prevention strategies and user training systems. These systems can be used either via a web browser on the client or through specific host-site software [8, 9]. Fig 2 presents the classification of Phishing detection approaches. Heuristic and ML based approach is based on supervised and unsupervised learning techniques. It requires features or labels for learning an environment to make a prediction. Proactive phishing URL detection is similar to ML approach. However, URLs are processed and support a system to predict a URL as a legitimate or malicious [11–15]. Blacklist and Whitelist approaches are the traditional methods to identify the phishing sites [16–21]. The exponential growth of web domains reduces the performance of the traditional method [22–24].

**Fig 2:** Anti—Phishing approaches.

The existing methods rely on new internet users to a minimum. Once they identify phishing website, the site is not accessible, or the user is informed of the probability that the website is not genuine. This approach requires minimum user training and requires no modifications to existing website authentication systems. The performance of the detection systems is calculated according to the following:

Number of True Positives (TP): The total number of malicious websites.
Number of True Negatives (TN): The total number of legitimate websites.
Number of False Positives (FP): The total number of incorrect predictions of legitimate websites as a malicious website.
Number of False Negatives (FN): The total number of incorrect predictions of malicious websites as a legitimate website.

Using some benchmark dataset, the accuracy of phishing detection systems is usually evaluated. The familiar phishing dataset to train the ML based techniques are as follows:

#### 2.2.1 Normal dataset

AlexaRank [25] is used as a benign and natural website benchmarking dataset. Alexa is a commercial enterprise which carries out web data analysis. It obtains the browsing habits of users from different sources and analyses them objectively for the reporting and classification of Internet web-based URLs. Researchers use the rankings provided by Alexa to collect a number of high standard websites as the normal dataset to test and classify websites. Alexa presents the dataset in the form of a raw text file where each line in the order ascended mentions the grade and domain name of a website.

#### 2.2.2 Phishing dataset

Phishtank is a familiar phishing website benchmark dataset which is available at https://phishtank.org/. It is a group framework that tracks websites for phishing sites. Various users and third parties send alleged phishing sites that are ultimately selected as legitimate site by a number of users. Thus, Phishtank offers a phishing website dataset in real-time. Researchers to establish data collection for testing and detection of Phishing websites use Phishtank’s website. Phishtank dataset is available in the Comma Separated Value (CSV) format, with descriptions of a specific phrase used in every line of the file. The site provides details include ID, URL, time of submission, checked status, online status and target URLs.

### 2.3 Research questions

Researcher framed the Research Questions (RQ) according to the objective of the study and its background. They are as follows:

RQ1—How URL detectors identify the phishing URLs or websites?
RQ2—How to apply ML methods to classify malicious and legitimate websites?
RQ3—How to evaluate a URL detector performance?

On the one hand, RQ1 and RQ2 assist to develop a ML based phishing detection system for securing an network from phishing attacks. On the other hand, RQ3 specifies the importance of the performance evaluation of a phishing technique. To address RQ1, authors found some recent literature related to URL detection using Artificial Intelligence (AI) techniques. The following part of this section presents the studies in detail with Table 2.

Authors in the study [2] proposed a URL-based anti-phishing machine learning method. They have taken 14 features of the URL to detect the website as a malicious or legitimate to test the efficiency of their method. More than 33,000 phishing and valid URLs in Support Vector Machine (SVM) and Naïve Bayes (NB) classifiers were used to train the proposed system. The phishing detection method focused on the learning process. They extracted 14 different features, which make phishing websites different from legitimate websites. The outcome of their experiment reached over 90% of precision when websites with SVM Classification are detected.

The study [3] explored multiple ML methods to detect URLs by analyzing various URL components using machine learning and deep learning methods. Authors addressed various methods of supervised learning for the identification of phishing URLs based on lexicon, WHOIS properties, PageRank, traffic rank information and page importance properties. They studied how the volume of different training data influences the accuracy of classifiers. The research includes Support Vector Machine (SVM), K-NN, random forest classification (RFC) and Artificial Neural Network (ANN) techniques for the classification.

Based on the output without and with the functionality selection a comparative study of machine learning algorithms is carried out in the study [4]. Experiments on a phishing dataset were carried out with 30 features including 4898 phished and 6157 benign web pages. Several ML methods were used to yield a better outcome. A method for selecting functions is subsequently employed to increase model performance. Random forests algorithm achieved the highest accuracy prior to and after the selection of features and dramatically increase building time. The results of the experiment shown that using the selection approach with machine learning algorithms can boost the effectiveness of the classification models for the detection of phishing without reducing their performance.

In this study [5], authors proposed URLNet, a CNN-based deep-neural URL detection network. They argued that current methods often use Bag of Words(BoW) such as features and suffered some essential limitations, such as the failure to detect sequential concepts in a URL string, the lack of automated feature extraction and the failure of unseen features in real—time URLs. They developed a CNNs and Word CNNs for character and configured the network. In addition, they suggested advanced techniques that were particularly effective for handling uncommon terms, a problem commonly exist in malicious URL detection tasks. This method can permit URLNet to identify embeddings and use sub word information from invisible words during testing phase.

Authors in [6] introduced a method for phishing URLs with innovative lexical features and blacklist. They collected a list of URLs using a crawler from URL repositories and collected 18 common lexical features. They implemented advanced ML techniques consisting of under/oversamples and classification. The automated approaches outperform other existing ML apporaches. The study has focused on content features and not lexical features, which was difficult to implement in real-world environments. The experimental results were better than the existing classification algorithms.

In the study [7], author investigated how well phishing URLs can be classified in the set of URLs which contain benign URLs. They discussed randomisation, characteristics engineering, the extraction of characteristics using host-based lexical analysis and statistical analysis. For the comparative study, several classifiers were applied and found that the results across the different classifiers are almost consistent. Authors argued that they proposed a convenient approach to remove functionality from URLs with simple standard words. More features could be experimented that lead to an optimum results. The dataset used in the study includes some older URLs. Thus, there is a possibility of lack of performance.

Authors [8] suggested a URL detector for high precision phishing attacks. They argued that the technique could be scaled to various sizes and proactively adapted. For both legitimate and malicious URLs a limited data collection of 572 cases had been employed. The characteristics were extracted and then weighed as cases to use in the prediction process. The test results were highly reliable with and without online phishing threats. For the improvement of the accuracy, Genetic algorithm (GA) has been used. Table 1 presents the outcome of the comparative study of literature.

**Table 1:** Comparison study of literature.

S. No.	Authors	Contributions	Limitations
1	Jain A.K., and Gupta B.B [2]	Employed both NB and SVM algorithms to identify the malicious websites.	Both SVM and NB are slow learners and does not store the previous results in the memory. Thus, the efficiency of the URL detector may be reduced.
2	Purbay M., and Kumar D. [3]	Utilized multiple ML methods for classifying URLs.	They compared the performance of different types of ML methods. However, there were no discussions about the retrieval capacity of the algorithms.
3	Gandotra E., and Gupta D. [4]	Applied multiple classification algorithms for detecting malicious URLs.	The outcome of the experiments demonstrated that the performance of the system was better rather than other ML methods. However, It lacks in handling larger volume of data.
4	Hung Le et al., [5]	Proposed a deep learning based URL detector. Authors argued that the method can produce insights from URL.	Deep learning methods demand more time to produce an output. In addition, it processes the URL and matches with library to generate an output.
5	Hong J. et al., [6]	Developed a crawler to extract URLs from data repositories. Applied lexical features approach to identify the phishing websites.	The performance evaluation was based on crawler-based dataset. Thus, there is no assurance for the effectiveness of the URL detector with real time URLs.
6	Kumar J. et al., [7]	Proposed a URL detector based on blacklisted dataset. Also, a lexical feature approach was employed to classify malicious and legitimate websites.	Authors employed an older dataset which can reduce the performance of the detector with real—time URLs.
7	Hassan Y.A. and Abdelfettah B. [8]	Suggested a URL detector for classifying websites and predict the phishing websites. They used GA technique to improve the performance.	The performance of GA based URL detector was better; nonetheless, the predicting time was huge with complex set of URLs.
8	Rao RS and Pais AR. [9]	Authors employed page attributes include logo, favicon, scripts and styles.	The method employed a server for updating the page attributes that reduces the performance of the detecting system.
9	Aljofey A et al. [10]	A CNN based detecting system for identifying the phishing page. A sequential pattern is used to find URLs.	The existing research shows that the performance of CNN is better for retrieving images rather than text.
10	AlEroud A and Karabatis G [11]	Generative adversarial network is used in the research to bypass a detection system.	Neural Network based detection system can identify the impression of an adverse network by learning the environment.

Authors [9] developed a detection approach for classifying malicious and normal webpages. The outcome of this study indicated that the value of true positive was higher rather than the false positive rate. In other study [10], authors proposed a Convolutional Neural Network (CNN) to detect a phishing URL. In this study, researchers employed a sequential pattern to capture the URL information. It achieved an accuracy of 98.58%, 95.46%, and 95.22%, respectively on benchmark datasets.

In study [11], authors employed a generative adversarial network for classifying the URLs and bypass the blacklist-based phishing detectors. In addition, researchers argued that the system can by pass both simple and novice ML detection techniques.

Based on the related work and its performance, authors selected a couple of studies for comparing with the proposed URL detector. The studies of Hung Le et al., [5] and Hong J. et al., [6] were selected. The reason for selecting studies is that the studies were applied deep learning methods and achieved an average accuracy of 90%.

## 3. Research methodology

RQ3 stated that how ML method can be employed to identify a malicious or legitimate URL. To present a solution, authors proposed a framework as shown in Fig 3 for classifying URLs and identify the phishing URLs.

**Fig 3:** Research framework.

Let $\sum_{n=0}^{m}x_{n}$ be the set of URLs where m is the maximum limit for the number (n) of URLs. Let M, L ∈ *x*_*n*_ be the malicious and legitimate, accordingly. Suppose M and L contains the properties Pm and Pl, respectively. The proposed framework employs RNN—LSTM to identify the properties Pm and Pl in an order to declare an URL as malicious or legitimate. The following equations from 1 to 4 presents the method for identifying the malicious URL. The term "recurring neural network" implies two broad groups of networks of a similar general structure, where one is a finite, and the other is an infinite input. Both network groups contains time dynamic behaviour. A recurrent network of finite input is a directed acyclic graph that can be replaced by a purely feedforward neural network, whereas a recurrent network of infinite input is a directed cyclical graph that cannot be modified. The modified version of RNN is LSTM. It is a deep learning method, which prevents the gradient problem of RNN. Multiple gates are employed for improving the performance of LSTM. In comparison with RNN, LSTM prevents back propagation. Each input of LSTM generates an output that becomes an input for the following layer or module of LSTM. Eqs 1 to 4 illustrates the concept of the proposed study.


$$\sum \left(M+L\right)=x_{n}$$ (1)

$$\text{Input}=\sum_{n=0}^{m}x_{n}$$ (2)

$$\text{Malicious}=\text{Output}\_\text{RNN}\left(\text{Input}\left(\text{Pm}\right)\right)$$ (3)

$$\text{Legitimate}=\text{Output}\_\text{RNN}\left(\text{Input}\left(\text{Pl}\right)\right)$$ (4)

During the training phase, RNN stores the properties Pm and Pl to learn the environment. Moreover, each URL of the dataset from Phishtank [23] and crawled URL is utilized in a way to instruct the model. Algorithm 3.1 and 3.2 presents the steps involved in the data collection and pre-process, correspondingly. Algorithm 3.3 and 3.4 shows the training phase and testing phase, individually. The training phase uses the labels to train RNN to learn the malicious and legitimate URLs. Thus, the testing phase of the proposed RNN model receives each URL and predicts the type of URL. RNN (LSTM) is developed with Python 3.0 in Windows 10 environment with the support of i7 processor.

LSTM model is an effective predictive model. It generates an output based on the arbitrary number of steps. There are five essential components that enables the model to produce long—term and short—term data.

Cell state (CS)—It indicates the cell space that accommodate both long term and short-term memories.

Hidden state (HS)—This is the output status information that user use to determine URL with respect to the current data, hidden condition and current cell input. The secret state is used to recover both short-term and long-term memory, in order to make a prediction.

Input gate (IT)—The total number of information flows to the cell state.

Forget gate (FT)—The total number of data flows from the current input and past cell state into the present cell state.

Output gate (OT)—The total number of information flows to the hidden state.

### 3.1. Input gate

It identifies an input value for memory alteration. Sigmoid defines the values that can be up to 0,1. And the tanh function weights the values passed by, evaluating their significance from-1 to 1. Eqs 5 and 6 represents the input gate and cell state, respectively. Wn is the weight, *HT*_*t*−1_ is the previous state of hidden state, *x*_*t*_ is the input, and *b*_*n*_ *is the bias vector* which need to be learnt during the training phase. CT is calculated using tanh function.


$$IT=\partial \left(W_{n}\left(HT_{t-1},x_{t}\right)+b_{n}\right)$$ (5)

$$CT=\text{tanh}(W_{d}\left(HT_{t-1},x_{t}\right)+b_{c})$$ (6)

### 3.2. Forget gate

It finds out the necessary block information to be discarded from the memory. The sigmoid function is used to describe it. Eq 7 contains (*HT*_*t*−1_) and content(*x*_*t*_) are examined, and the number of outputs between 0 and 1 is verified by each cell state *CT*_*t*−1_ number.


$$FT=\partial \left(W_{f}\left(HT_{t-1},x_{t}\right)+b_{f}\right)$$ (7)

### 3.3. Output gate

The input and the memory of the block is used to determine the output. Sigmoid function determines which values to let through 0 and 1. The tanh function presents weightage to the values which are transferred to determine their degree of importance ranging from-1 to 1 and multiplied with output of Sigmoid.


$$OT=\partial \left(W_{o}\left(HT_{t-1},x_{t}\right)+b_{o}\right)$$ (8)

$$HT=O_{t}*\text{tanh}\left(C_{t}\right)$$ (9)

Fig 4 represents the processes involved in data collection. Data Repositories such as Phishtank and Crawler are used to collect Malicious and Benign URLs. A crawler is developed in order to collect URLs from AlexaRank website. AlexaRank publishes set of URLs with ranking to support to research community. In this study, the crawler crawled a number of 7658 URLs from AlexaRank between June 2020 to November 2020. 6042 URLs were collected through Phishtank datasets. During the data collection, extracted data are stored in W and returned as W1 with number of URLS, N.

**Fig 4:** Algorithm—Data collection.

Fig 5 illustrates the steps of data pre—process. url is one of the elements of URL dataset. In this process, the raw data is pre—processed by scanning each URL in th dataset. A set of functions are developed in order to remove the irrelevant data. Finally, D2 is the set of features returned by the pre—process activity.

**Fig 5:** Algorithm—Data pre-process.

Fig 6 represents the processes of data transformation. “Num” is the vector returned by the data transformation process. During this process, each feature of D2 is converted as a vector. Each data in D2 is processed using the GenerateVectors function. A vector is generated and passed as an input to the training phase.

**Fig 6:** Algorithm—Data transformation.

Fig 7 provides the processes involved in the training phase. Each URL is processed with the support of vector. LSTMLib is one of the functions in the LSTM to predict an output using the vectors. The library is updated with the extracted features that contains the necessary data related to malicious and normal web pages. Thus, the iterative process is used to scan each vector and suspicious URL and generate a final outcome. Lastly, op is the prediction returned by the proposed method during the training phase.

**Fig 7:** Algorithm—Training phase.

Fig 8 indicates the testing phase of the proposed URL detection. The proposed processes each element from LSTMMemory function is compared with the vector of URL and decide an output. The f is the element of the feedback which is collected from the crawler that indicates the page rank of a website. The page rank indicates the value of a website and the lowest ranking website will be declared as malicious or suspicious to alert the users.

**Fig 8:** Algorithm—Testing phase.

Fig 9 shows the snippet of epoch settings in the training phase. The epoch value is used to indicate the execution time of a method. The learning rate can be increased to improve the performance of a method.

**Fig 9:** Epoch settings—Training phase.

## 4. Results and discussions

The proposed method (LURL) is developed in Python 3.0 with the support of Sci—Kit Learn and NUMPY packages. Also, the existing URL detectors are constructed for evaluating the performance of LURL. Table 2 shows the parameters settings of methods during training and testing phases. Learning rate, maximum epoch, batch size, and decay are the parameters to instruct the methods to execute the results for certain number of times. Threshold values and vocabulary size are the important parameters for testing phase to generate results using test dataset.

**Table 2:** Initial settings of parameters (training and testing phases).

Methods	Training phase	Testing phase
LURL	learning_rate = 1.0, max_lr_epoch = 7, lr_decay = 0.73batch_size = 2, num_steps = 31, data = train_data	batch_size = 20, num_steps = 35, data = test_datanum_acc_batches = 30, check_batch_idx = 25, acc_check_thresh = 5, s_training = False, hidden_size = 650, vocab_size = vocabulary, num_layers = 2
Hung Le et al.,	learning_rate = 1.0, max_lr_epoch = 9, lr_decay = 0.42, batch_size = 2, num_steps = 31, data = train_data	batch_size = 20, num_steps = 35, data = test_datanum_acc_batches = 30, check_batch_idx = 21, acc_check_thresh = 6, s_training = False, hidden_size = 700, vocab_size = vocabulary, num_layers = 2
Hong J. et al.,	learning_rate = 1.0, max_lr_epoch = 9, lr_decay = 0.93, batch_size = 2, num_steps = 31, data = train_data	batch_size = 20, num_steps = 35, data = test_datanum_acc_batches = 30, check_batch_idx = 22, acc_check_thresh = 6, s_training = False, hidden_size = 750, vocab_size = vocabulary, num_layers = 2

The methods are evaluated in terms of learning rate, accuracy, and precision. Table 3 presents the learning rate of the methods during the training phase. The performance of three detectors during the training phase are similar. It is evident that the learning ability of methods are same. Authors maintained similar parameters for all detectors. However, the proposed method, LURL produced a better outcome rather than Hung Le et al. [5] and Hong J. et al. [6]. LURL covered 94.3 percent of data with learning rate of 5.0 whereas Hung Le et al. and Hong J. et al. have reached 93.8 and 92.8, respectively. The learning rate of LURL is reasonable comparing to other two methods. It indicates that ML based methods able to scan an average of 84% of dataset to learn the environment at the rate of 1.0.

**Table 3:** Learning rate—Performance comparison with Phishtank dataset.

Learning Rate	LURL	Hung Le et al.	Hong J. et al.
1.0	*86*.*3*	83.6	85.4
2.0	*89*.*5*	88.9	87.9
3.0	*92*.*1*	90.7	91.3
4.0	*91*.*6*	92.4	91.8
5.0	*94*.*3*	93.8	92.8

Table 4 shows the learning rate of the methods for Crawler dataset. As discussed in the section 3, Crawler dataset was generated with the support of AlexaRank dataset. It contains larger number of normal URLs comparing to the malicious URLs. The intention for employing Crawler is to teach the methods to predict legitimate URLs. It is very difficult to predict a website without analysing content; however, the phishing site is similar to legitimate website. Therefore, it is necessary for methods to understand the differences between legitimate and malicious website. Based on the outcome, it is obvious that the performance of all detectors is like each other. Similar to Phishtank dataset, all three methods consumed an average of 86% of data at the rate of 1.0. The reason for the faster rate is that RNN can read numeric data at faster rate rather than images [12].

**Table 4:** Learning rate—Performance comparison with Crawler dataset.

Learning Rate	LURL	Hung Le et al.	Hong J. et al.
1.0	*87.5*	86.8	89.7
2.0	*89.2*	88.1	89.6
3.0	*90.6*	91.3	90.3
4.0	*91.7*	90.8	91.8
5.0	*93.6*	92.4	94.1

There is a demand for an effective phishing detection system to secure a network or individual’s privacy and data. RQ3 supports to evaluate the performance of the proposed method using the learning rate, accuracy, and F1 score. RQ3 states that how to measure the efficiency of URL detectors. Tables 5 and 6 presents a solution for it. Table 5 shows the accuracy of detectors with Phishtank and Crawler datasets, accordingly. LURL has produced an average of 97.4% and 96.8% for Phishtank and Crawler datasets respectively. Both Hung Le et al., and Hong J. et al., have reached an average of 93.8, 94.1, 96.7, and 93.6 for Phishtank and Crawler datasets. It is evident that the performance of LURL is better comparing to other URL detectors. Fig 10 illustrates the corresponding graph of Table 4. It represents that LURL has generated the output in less amount of time rather than the other predictors.

**Fig 10:** Accuracy of Phishtank and Crawler dataset.

**Table 5:** Comparison of accuracy.

Methods	Phishtank		Crawler	
	Accuracy (%)	Time (in Seconds)	Accuracy (%)	Time (in Seconds)
LURL	*97*.*4*	*3*.*45*	*96*.*8*	*4*.*21*
Hung Le et al.	93.8	5.12	94.1	4.79
Hong J. et al.	96.7	4.78	93.6	3.79

**Table 6:** Comparison of F1—Measure.

Methods	Phishtank		Crawler	
	F1- Score	Time (in Seconds)	F1—Score	Time (in Seconds)
LURL	*96*.*4*	*4*.*62*	*96*.*2*	*3*.*89*
Hung Le et al.	95.8	3.87	95.6	4.91
Hong J. et al.	92.7	5.23	95.3	3.62

Finally, Table 6 provides the comparison of F1—score of URL detectors. As presented in section 2, TP and TN indicate the malicious and legitimate URLs, accordingly. Based on the TP, TN, FP, and FN, both precision and recall value are calculated. Using these values, F1—measure is computed. It indicates the retrieving ability of URL detector. From the outcome, it is obvious that the proposed URL detector, LURL is superior rather than other two URL detectors. The reason for the better F1—measure is the capability of LSTM memory. Fig 11 shows the F1—score against the computation time. It represents that LURL achieved a F1—Score of 96.4 in 4.62 seconds for Phishtank dataset whereas Hung Le et al., and Hong J. et al., have achieved 95.8, 92.7 in 3.87 and 5.23 respectively. For Crawler dataset, F1—Score of LURL is 94.8 whereas Hung Le et al. and Hong J. et al. has reached 95.6, and 95.3, accordingly.

**Fig 11:** F1—Score of Phishtank and Crawler dataset.

## 5. Conclusion

The proposed study emphasized the phishing technique in the context of classification, where phishing website is considered to involve automatic categorization of websites into a predetermined set of class values based on several features and the class variable. The ML based phishing techniques depend on website functionalities to gather information that can help classify websites for detecting phishing sites. The problem of phishing cannot be eradicated, nonetheless can be reduced by combating it in two ways, improving targeted anti-phishing procedures and techniques and informing the public on how fraudulent phishing websites can be detected and identified. To combat the ever evolving and complexity of phishing attacks and tactics, ML anti-phishing techniques are essential. Authors employed LSTM technique to identify malicious and legitimate websites. A crawler was developed that crawled 7900 URLs from AlexaRank portal and also employed Phishtank dataset to measure the efficiency of the proposed URL detector. The outcome of this study reveals that the proposed method presents superior results rather than the existing deep learning methods. A total of 7900 malicious URLS were detected using the proposed URL detector. It has achieved better accuracy and F1—score with limited amount of time. The future direction of this study is to develop an unsupervised deep learning method to generate insight from a URL. In addition, the study can be extended in order to generate an outcome for a larger network and protect the privacy of an individual.

## Supporting information

S1 File (ARFF)

S1 Data (CSV)
